# Plumbagin Ameliorates Diabetic Nephropathy via Interruption of Pathways that Include NOX4 Signalling

**DOI:** 10.1371/journal.pone.0073428

**Published:** 2013-08-26

**Authors:** Rachel Yong, Xin-Ming Chen, Sylvie Shen, Swarna Vijayaraj, Qing Ma, Carol A. Pollock, Sonia Saad

**Affiliations:** Department of Medicine, Kolling Institute of Medical Research, Northern Clinical School, University of Sydney, Sydney, Australia; UCL Institute of Child Health, United Kingdom

## Abstract

NADPH oxidase 4 (Nox4) is reported to be the major source of reactive oxygen species (ROS) in the kidneys during the early stages of diabetic nephropathy. It has been shown to mediate TGFβ1-induced differentiation of cardiac fibroblasts into myofibroblasts. Despite TGFβ1 being recognised as a mediator of renal fibrosis and functional decline role in diabetic nephropathy, the renal interaction between Nox 4 and TGFβ1 is not well characterised. The aim of this study was to investigate the role of Nox4 inhibition on TGFβ1-induced fibrotic responses in proximal tubular cells and in a mouse model of diabetic nephropathy. Immortalised human proximal tubular cells (HK2) were incubated with TGFβ1 ± plumbagin (an inhibitor of Nox4) or specific Nox4 siRNA. Collagen IV and fibronectin mRNA and protein expression were measured. Streptozotocin (STZ) induced diabetic C57BL/6J mice were administered plumbagin (2 mg/kg/day) or vehicle (DMSO; 50 µl/mouse) for 24 weeks. Metabolic, physiological and histological markers of nephropathy were determined. TGFβ1 increased Nox4 mRNA expression and plumbagin and Nox4 siRNA significantly inhibited TGF-β1 induced fibronectin and collagen IV expression in human HK2 cells. STZ-induced diabetic C57BL/6J mice developed physiological features of diabetic nephropathy at 24 weeks, which were reversed with concomitant plumbagin treatment. Histologically, plumbagin ameliorated diabetes induced upregulation of extracellular matrix protein expression compared to control. This study demonstrates that plumbagin ameliorates the development of diabetic nephropathy through pathways that include Nox4 signalling.

## Introduction

Understanding the mechanisms of tubulointerstitial fibrosis is essential for the establishment of novel therapeutic strategies for the prevention or arrest of progressive kidney disease. Transforming growth factor-beta is considered a critical fibrogenic factor [1]. Under pathological conditions, TGF-β_1_ is amplified and correlates with clinical and histological markers of progressive pathology [2]. However, targeting of TGFB to reduce nephropathy has not been uniformly successful, largely due to its pleotrophic effects.

NADPH oxidase 4 (Nox4) is a constitutively active multisubunit enzyme, which generates superoxide from molecular oxygen using NADPH as the electron donor. It acts as an oxygen sensor, catalyzing the reduction of molecular oxygen to various reactive oxygen species (ROS). Nox4 is widely expressed in the kidney [3]. It has been reported that Nox4 is the major source of ROS in the kidneys during the early stages of diabetes mellitus and Nox4-derived ROS are considered to mediate renal hypertrophy, increase fibronectin expression [4] and myofibroblast activation induced by TGFβ1 [5]. ROS are increasingly recognized as playing a major role in upregulating intracellular signaling molecules with the end result being renal fibrosis [6], [7], [8], [9]. ROS transduce and amplify glucose signalling in renal cells in high glucose environments and play a critical role in excessive extracellular matrix (ECM) deposition in the diabetic kidney. Both ROS and TGF β1 are induced in hyperglycaemic conditions. Nox4 has been shown to mediate TGFβ1-induced differentiation of cardiac fibroblasts into myofibroblasts [10] and proliferation of human pulmonary artery smooth muscle cells [11]. Nox4 deficiency and acute inhibition of Nox4 prevents TGF-β1-induced cell death in primary alveolar epithelial cells [12]. Nox4 has recently been shown to be implicated in glucose induced oxidative stress in the kidney and in profibrotic processes in renal cells [13]. However, the role of Nox4 in TGFβ1 mediated fibrotic responses in the kidney, and particularly in human proximal tubule cells, the most prominent cell type in the renal cortex which influences fibrotic processes, is not known. In this study we hypothesise that targeting Nox4 in diabetes mellitus will decrease ROS generation and mitigate the development of renal pathology. The proposed studies will provide ‘proof of concept’ that targeting Nox4 will attenuate, or reverse the development of renal fibrosis in patients with diabetes mellitus**.**

## Materials and Methods

### 1. Ethics Statement

Experiments in this study were approved by the Animal Care and Ethics Committee of Royal North Shore Hospital and were performed according to the recommendations of the Australian Council for Animal Care.

### 2. Cell Culture

Human kidney-2 (HK-2) cells, an immortalized human kidney proximal tubule cell line from American Type Cell Collection (ATCC, USA), were used in this study. Cells were grown in keratinocyte serum-free media (KSFM) (Invitrogen, USA) and seeded at 80–90% confluence prior to exposure to 5 mM d-glucose (normal glucose) or 2 ng/ml TGFβ1 in the presence and absence of 1 µM of plumbagin (Nox4 inhibitor) [14], [15] for either 24 or 48hrs. We have demonstrated that Plumbagin has an IC 50 for Nox4 of 0.5 µM. Cell viability assays using 0.5 or 1 µM showed no cell toxicity (data not shown). Given the lack of specificity of any pharmacological inhibitor of Nox 4, including Plumbagin, the role of Nox4 was determined using specific siRNA studies targeting Nox4 mRNA as discussed below. Supernatants were reserved for Western blot analysis and RNA was extracted for real time PCR.

### 3. In vivo Experiments

Streptozotocin (STZ)-induced diabetes mellitus in a mouse C57BL/6J model was used for these studies due to its reproducibility and low toxicity with multiple low dosage injections. Briefly, the inbred male C57BL/6J mice (8 weeks, 21–26 g) were maintained under standard animal house conditions. Mice were given intraperitoneal injections of STZ (Sigma-Aldrich) in sodium citrate buffer (pH 4.5) on 5 consecutive days (55 mg/kg/day). To test whether the Nox4 inhibitor plumbagin attenuates renal fibrosis in the diabetic mice, the following three groups (16 mice per group) were studied: (1) non-diabetic control +DMSO; (2) diabetic + DMSO; (3) diabetic + plumbagin. After 5 STZ injections, mice were treated with i.p.-injections of the Nox4 blocker plumbagin (2 mg/kg/day) as previously described [16], [17] or vehicle (DMSO) daily. Blood sugar level, blood pressure, plasma creatinine, microalbuminuria and creatinine clearance were assessed weekly. The animals were sacrificed at 24 wks after STZ administration, blood was collected and both kidneys harvested for real time PCR or immunohistochemistry.

### 4. Plasma and urine measurements

A 24 hr urine and blood obtained from cardiac puncture in the three experimental groups were collected at the study end point. Levels of plasma glucose were determined using an automated analyser (Synchron CX5 PRO; Beckman). Creatinine clearance and albuminuria were measured using enzyme-linked immunosorbent assay (Albuwell and Creatinine companion kit; Exocell, Philadelphia, PA) according to the manufacturer’s instructions.

### 5. TGFβ1 ELISA

Cells were seeded at 2×10^5^ cells/well in a 24-well plate and grown in KSFM in the absence of growth factors for 24 h. At 70% confluence, cells were exposed to the experimental conditions as defined above for 48 h in quadruplicate. Supernatants were then collected, spun, and stored at −20°C until TGF-β_1_ levels were determined by immunoassay (Promega) as per the manufacturer’s instructions. Cell lysate protein concentration was determined (Bio-Rad), and TGF-β_1_ levels were corrected for protein content per well.

### 6. Western Blotting

HK2 cells supernatants from the above culture conditions were collected and equal amounts were resolved on 7.5% SDS-PAGE electrophoresis. Proteins were then blotted on a nitrocellulose membrane. Fibronectin (Sigma Aldrich) or Collagen IV (Abcam) antibodies (1/1000 each) were used overnight followed by incubation with anti rabbit or anti mouse antibody (Amersham Pharmaceuticals) for 1 hr at room temperature. The bands corresponding to fibronectin (220 KDa) or collagen IV (200 KDa) were quantified using NIH Image soft v1.60. Equal protein loading was confirmed using coomassie blue staining (Biorad) for 2 hrs followed by destaining solution (Biorad) for 1 hrs. Data were adjusted and expressed as percentage of control.

### 7. Nox4 Silencing

To complement pharmacological inhibition of Nox4, siRNA was designed to specifically target Nox4 mRNA. Nox4 siRNA sequence is as follow: GCAGGAGAACCAGGAGAUU' (Ambion). HK2 cells were transfected with 8 nM Nox4 siRNA using Lipofectamine (Invitrogen) as per manufacturer’s instructions. Cells were then exposed to the above culture conditions for 48 hrs. Cells were collected to determine fibronectin and collagen IV mRNA levels by real time PCR. All siRNA experiments included non-specific control (NSC siRNAs, Ambion). Nox4 knockdown was confirmed by real time PCR.

### 8. RT- PCR

Total RNA was extracted from either HK2 cells or kidney tissues using the TRIzol method (Invitrogen). Quantitative real-time PCR (TaqMan; Roche Molecular Diagnostics) was used to measure the expression of fibronectin, collagen IV, Nox4, TGFβ1 and superoxide dismutase -1 (SOD1). Data were expressed relative to the housekeeping gene GAPDH or Actin. Human and mice primer sequences are detailed in Table 1.

**Table 1:** Primer sequences for human (h) and mice (m).

Gene	Primer Sequences
h Fibronectin	Forward: 5′-GCGAGAGTGCCCCTACTACA-3′
	Reverse: 5′-GTTGGTGAATCGCAGGTCA-3′
h Collagen	Forward: 5′-CGGGTACCCAGGACTCATAG-3′
	Reverse: 5′-GGACCTGCTTCACCCTTTTC-3′
h GAPDH	Forward: 5′-AGCCACATCGCTCAGACAC-3′
	Reverse: 5′-GCCCAATACGACCAAATCC-3′
h Nox4	Forward: 5′-CTTTTGGAAGTCCATTTGAG-3′
	Reverse: 5′-CGGGAGGGTGGGTATCTAA-3′
h SOD1	Forward: 5′-AAGTACAAAGACAGGAAACG-3′
	Reverse: 5′-AGCAACTCTGAAAAAGTCAC-3′
m NoX4	Forward: 5′-CTGGTCTGACGGGTGTCTGCATGGTG-3′
	Reverse: 5′-CTCCGCACAATAAAGGCACAAAGGTCCAG-3′
m SOD1	Forward: 5′-GGTGAACCAGTTGTGTTGTCAGG-3′
	Reverse: 5′- ATGAGGTCCTGCACTGGTACAG-3′
m TGF-β1	Forward: 5′-TCAGACATTCGGGAAGCAGT-3′
	Reverse: 5′-ACGCCAGGAATTGTTGCTAT-3′
m Fibronectin	Forward: 5′-CACGGAGGCCACCATTACT-3′
	Reverse: 5′-CTTCAGGGCAATGACGTAGAT-3′
m Collagen IV	Forward: 5′-TTAAAGGACTCCAGGGACCAC-3′
	Reverse: 5′-CCCACTGAGCCCTGTCACAC-3′
m β-Actin	Forward: 5′-CCCACTGAGCCCTGTCACAC-3′
	Reverse: 5′-GTGGTACGACCAGAGGCATAC-3′

### 9. Superoxide Dismutase Assay

Total SOD activity in tissue homogenates was determined using the Superoxide Dismutase Assay Kit II (Calbiochem) according to the manufacturer’s instructions. This assay utilizes a tetrazolium salt for detection of superoxide radicals generated by xanthine oxidase and hypoxanthine. One unit of SOD was defined as the amount of enzyme needed to exhibit 50% dismutation of the superoxide radical. Data were adjusted/protein concentration and expressed as units/mg protein.

### 10. Renal structure and Immunohistochemistry

Kidneys were fixed in 4% paraformaldehyde (PFA) and paraffin embedded sections (4 µM thickness) were prepared. Sections were stained with periodic acid Schiff’s and Masson’s Trichrome and examined by light microscopy. For immunohistochemistry, sections were incubated with primary antibodies against proliferating cell nuclear antigen (PCNA) (SantaCruz), fibronectin (Sigma Aldrich), 8-hydroxy-deoxyguanosine (8-OHdG) (Bioss), Nox4 (Santacruz) and nitrotyrosine (Upstate) using a sequenza vertical cover-plate immunostaining system overnight at 4°C. Detection was performed using horseradish peroxidase anti-rabbit Envision + system with diaminobenzidine (Dako). Sections were then counterstained with hematoxylin. Epitope retrieval was performed using 0.01 M Citrate buffer pH 6.0 by a pressure cooker set at 121°C for 30 sec. Control sections were also prepared in which the authentic primary antibodies were replaced with an irrelevant isotype matched IgG. The tissue specimens were examined by bright field microscopy using a Leica photomicroscope linked to a DFC 480 digital camera.

### 11. Quantitation of histological parameters

In brief, 10 random non-overlapping fields from three stained sections were captured. Digitised images were then loaded onto a Pentium D Dell computer. Areas of brown staining reflecting PCNA, Nitrotyrosine, 8-OHdG, Nox4 and fibronectin expression were highlighted using a selective colour tool for their colour ranges, and the proportional area of the tissue with their respective ranges of colour was then quantified. Calculation of the proportional area stained brown was then determined using the automated cellular imaging system ACIS III (Dako).

Glomerulosclerosis was quantified on PAS-stained sections employing a score of 0–4 as described by Hartner *et al*. [18]. Twenty glomeruli per cross-section were evaluated for glomerulosclerosis. Assessment was done in a blinded fashion by two researchers independently. A relative quantitation was also performed on marked glomeruli using the ACIS III program and data was expressed relative to control.

Masson trichrome-stained sections were used for morphometric analysis of interstitial fibrosis. The percentage of blue-stained area in digitized images was quantitated using ACIS III. A total of 12–20 images per section were evaluated after marking non-tubulointerstitial areas (glomeruli, tubular and vascular lumen, artefacts) that were excluded from analysis.

### 12. Statistical Analysis

All *in vitro* results are expressed as a percentage of the control value. Experiments were performed in at least three different culture preparations, and at least three data points for each experimental condition were measured in each preparation. Results are expressed as mean ± SEM, with *n* reflecting the number of culture preparations. Statistical comparisons between groups for in vitro and in vivo data were made by analysis of variance (anova), with pairwise multiple comparisons made by Fisher's protected least-significant difference test using the software package Statview v4.5 (Abacus Concepts, CA, USA) values ≤0.05 were considered significant.

## Results

### 1. High glucose and TGF-β1 increase Nox4 mRNA expression

We have previously demonstrated that high glucose increases the profibrotic marker TGFβ production in HK2 cells to 138±6.5% (P<0.05 vs control) [19]. We have additionally demonstrated that high glucose increases TGFβ mRNA expression to 1.4±0.26 fold (P<0.05 vs control) and Nox4 mRNA expression to 2.76±0.47 fold (P<0.05 vs control) (Fig 1 A,B and C). In addition, we have shown that TGF-β1 increases Nox4 mRNA expression to 2.8±0.5 fold (P<0.05 vs control). This suggests a role for Nox4 in mediating high glucose effect and downstream effects of TGF-β1 in the proximal tubule.

**Figure 1:** High glucose and TGF-β1 induced Nox4 expression. A) Real time PCR showing increased TGF β1 mRNA expression in high glucose treated HK2 cells. B) ELISA showing TGF β1 levels in pg/ml of protein produced following exposure of HK2 cells to high glucose. Real time PCR showing Nox4 mRNA expression following exposure to high glucose (C) or TGF-β1 (D). HK2 were incubated for 24 hrs with 5 mM glucose media (control), 30 mM D glucose or TGF-β1 (2 ng/ml). Data is normalised by glyceraldehyde-3-phosphate dehydrogenase (GAPDH) and expressed as mean ± SEM; n = 3. *P<0.05 vs. Control.

### 2. Plumbagin reverses the effect of TGF-β1 on SOD1 mRNA expression

Plumbagin, a pharmacological inhibitor of Nox4, had no effect on Nox4 mRNA expression or TGFβ mediated Nox4 increased mRNA expression as expected (Fig 2A). Since Nox4 is the major source of ROS in the kidneys during the early stages of diabetic nephropathy and in order to confirm the effect of TGFβ1 on ROS production, the levels of SOD1, which constitutes the first line of defence against ROS were determined following TGFβ1 treatment. We have clearly demonstrated that TGF-β1 significantly reduced SOD1 mRNA expression to 0.66±0.1 fold (P<0.05 vs control). Conversely, plumbagin increased SOD1 expression to 1.7±0.3 fold (P<0.05 vs control) (Fig 2B).

**Figure 2:** Plumbagin effect on Nox4 and SOD1 mRNA levels. HK2 were incubated for 24 hrs with 5 mM glucose media (control); Plumbagin (Plg) or TGF-β1 ± Plg in control media. A) Nox4 mRNA expression normalised by GAPDH. B) Normalized SOD1 mRNA expression. Results are expressed as mean ± SEM; n = 4. * *P*<0.05 vs. control.

### 3. Plumbagin inhibits TGF-β1 induced fibronectin and collagen IV mRNA expression

Fibronectin and collagen IV are major extracellular matrix proteins that serve as a scaffold for the deposition of other proteins. Upregulation of fibronectin and collagen IV are regarded as markers of tubulointerstitial fibrosis. As expected, TGF-β1 induced fibronectin and collagen IV mRNA expression in HK2 cells to 1.3±0.04 fold and 1.5±0.08 fold respectively (both P<0.005 vs control). In order to determine the dependency of ECM protein upregulation on Nox4, Nox4 inhibitor (Plumbagin) was used in the presence and absence of TGF-β1. Plumbagin blocked TGF-β1 induced upregulation of fibronectin and collagen IV mRNA levels to 0.85±0.05 fold and 0.96±0.1 fold respectively; (both P<0.005 vs TGF-β1; Fig 3).

**Figure 3:** Plumbagin blocked TGF-β1 induced fibronectin and collagen IV mRNA levels. HK2 were incubated for 24 hrs with 5 mM glucose media (control); Plumbagin (Plg) or TGF-β1 ± Plg in control media. A) Fibronectin mRNA expression normalised by GAPDH. B) Normalized collagen IV mRNA expression. Results are expressed as mean ± SEM; n = 4. *#P*<0.005 vs. control or indicated experimental conditions.

### 4. Plumbagin inhibitsTGF-β1 induced fibronectin and collagen IV protein production

TGF-β1 similarly increased fibronectin and collagen IV protein production to 318± 79% (P<0.05) and 249±54% (P<0.005) respectively. Plumbagin was able to completely reverse the stimulated production of fibronectin protein to 103± 28% (P<0.05 vs TGF-β1) and of collagen IV to 67±17% (P<0.005 vs TGF-β1). Plumbagin of itself has no effect on fibronectin and collagen IV production (Fig 4 A and B).

**Figure 4:** Plumbagin blocked TGF-β1 induced fibronectin and collagen IV protein levels. HK2 were incubated for 48 hrs with 5 mM glucose media (Control); Plumbagin (Plg) or TGF-β1 ± Plg in control media. A) Representative Western blotting images for fibronectin and coomassie blue protein stain and normalized results expressed as mean ± SEM; n = 3. *P<0.05 vs. control or indicated experimental conditions. B) Representative Western blotting images for collagen IV and coomassie blue protein stain and normalized results expressed as mean ± SEM; n = 4. *#P*<0.005 vs. Control or indicated experimental conditions.

### 5. Nox4 siRNA significantly inhibits Nox4 mRNA expression and reverses TGF-β1 effect on Nox4 and SOD 1 expression

Since plumbagin has known non specific effects and in order to confirm the role of Nox4 in TGFβ mediated effects, specific Nox4 siRNA was used. We have shown that Nox4 siRNA significantly inhibited Nox4 mRNA expression to 0.2±0.02 fold (P<0.0001 vs NSC) Fig 5A, and increases SOD1 expression to 1.5±0.24 fold (P<0.05 vs NSC) Fig 5B. Nox4 siRNA significantly reversed TGF-β1 effect on Nox4 and SOD1 mRNA expression to 0.8±0.1 fold and 1.2±0.1 fold respectively (Fig 5 A and B).

**Figure 5:** Effect of Nox4 siRNA on TGF-β1 mediated effect on Nox4 and SOD1 expression. Real time PCR showing Nox4 mRNA expression (A) and SOD1 mRNA expression (B) following TGF-β1 exposure in the presence of non specific control siRNA (NSC) or Nox4 siRNA for 24 hrs. Data is normalised by GAPDH and expressed as mean ± SEM; n = 3. * *P<*0.05 and *#P*<0.0005 and ** *P*<0.0001 vs. control or indicated experimental conditions.

### 6. Nox4 siRNA inhibits TGF-β1 induced fibronectin and collagen IV mRNA expression

Using Nox4 siRNA, we confirmed that both TGF-β1 mediated induction of fibronectin and collagen IV were significantly reduced to 0.5±0.1 fold (P<0.005) and 2.5±0.08 fold (P<0.05) versus TGF-β1 respectively (Fig 6 A and B). This confirms that TGF-β1 mediated upregulation of extracellular matrix involves the Nox4 pathway

**Figure 6:** Nox4 siRNA blocks TGF-β1 induced fibronectin and collagen IV mRNA levels. HK2 were incubated for 24 hrs with scrambled non specific control (NSC) in 5 mM glucose media; TGF-β1 ± NSC or Nox4 siRNA in control media. A) Fibronectin mRNA expression normalised by glyceraldehyde-3-phosphate dehydrogenase (GAPDH). B) Normalized collagen IV mRNA expression. Results are expressed as mean ± SEM; n = 4. *#P*<0.005 and *P<0.05 vs. control or indicated experimental conditions.

### 7. Nox4 expression and ROS production increases in the kidneys of diabetic mice and are reduced by administration of the Nox4 inhibitor plumbagin

We have shown that Nox4 is expressed in C57BL/6J control kidney in the proximal and distal tubules at low levels and its level was significantly increased in the diabetic kidney (Fig 7B) compared to control (7A). Since Nox4 is the major source of ROS production in the kidneys during the early stages of diabetes, the level of nitrotyrosine, as a marker of ROS production [20] and the levels of 8-OHdG, as a marker for ROS induced DNA damage, were determined in diabetic mice in the presence and absence of plumbagin. Our data showed that kidneys from diabetic mice express increased levels of nitrotyrosine and 8-OHdG in their tubules, suggestive of increased ROS production (Fig 7E and H) compared to control (7D and G). Plumbagin administration significantly blocked diabetic induced Nox4 expression (Fig 7C) nitrotyrosine and 8-OHdG expression (Fig 7F and I respectively). Increased levels of Nox4 mRNA and reduced levels of SOD1 mRNA were additionally shown in the diabetic mice to 2.6±0.26 fold and 0.4±0.1 fold P<0.05 vs control both (Fig 8 A and B). Interestingly Nox4 and SOD1 effects were reversed by plumbagin administration to 0.75±0.1 fold (P<0.05 vs diabetic) and 1.07±0.2 fold (P<0.05 vs diabetic) respectively (Fig 8A and B). In addition, SOD activity was significantly reduced in the diabetic animals to 51±8.8% (P<0.05vs control) (Fig 8C). Plumbagin significantly increased SOD activity when it was administered to the diabetic animals to 194.6±5.1% (P<0.05 vs control and P<0.005 vs diabetic) suggesting an antioxidant effect (Fig 8C).

**Figure 7:** Nox4 expression and ROS production *in vivo*. Immunohistochemistry demonstrating that Nox4, nitrotyrosine and 8-OHdG protein expression are highly expressed in STZ-induced diabetic C57BL/6J mice (B, E and H respectively) compared to controls (A, D and G). Plumbagin (2 mg/kg/day) administration blocked diabetic induced Nox4, nitrotyrosine and 8-OHdG expressions (C, F and I). Proportion of area immunostained for Nox4, nitrotyrosine and 8-OHdG are shown (J, K, L). STZ and plumbagin were administered as described in the Material and Methods. Negative IgG was performed to confirm staining specificity (not shown). Magnification x 400.

**Figure 8:** Expression of oxidative stress markers, Nox4 and SOD1 in diabetic mice in the presence and absence of plumbagin. A) Nox4 mRNA expression normalised to Actin. B) Normalized SOD1 mRNA expression. C) SOD activity expressed as unit/mg of protein. Results are expressed as mean ± SEM; n = 5-7. *#P*<0.005 and *P<0.05 vs. control or indicated experimental conditions.

### 8. Nox4 inhibition improves renal physiological markers in mice with diabetes mellitus

The data detailed in Table 2 clearly confirms that STZ-induced diabetes mellitus in C57BL/6J mice induces renal physiological features of diabetic nephropathy at 24 weeks which are reversed with concomitant plumbagin treatment. Diabetic animals demonstrated increased serum creatinine levels to 25±4% µmol/l vs non diabetic control (13 ±1%; P = 0.001), increased urine albumin/creatinine ratio to 13.2±1.5 vs 3.4±0.4 mg/mmol (P<0.0005), increased kidney to body weight to 9.55±0.4×10^−3^ vs 6.9±0.2×10^−3^ g/g (P<0.0001) and increased 24 hr urine output compared to non diabetic control mice to 6.5±2.4 vs 0.7+0.1 ml respectively P = 0.005. Creatinine clearance rate was also reduced in STZ induced diabetic mice compared to non diabetic controls 1.56±4×10^−4^ vs 2±6×10^−4^ ml/min respectively. These data collectively suggest improved kidney function with Nox4 inhibition.

**Table 2:** Physiological markers in diabetic mice in the presence and absence of plumbagin.

	Non Diabetic (i)	Diabetic-DMSO (ii)	Diabetic-Nox4 inhibitor iii	P value (ii vs i)	P value (iii vs i)	P value (iii vs ii)
Serum Creatinine (µmol/L)	13.3±1.2	25.3±4.0^#^	14.8±1.1^#^	0.001	0.55	0.004
Cr Clearance Rate (ml/min)	2.0±6.2×10^4^	1.56±4.0×10^4^	1.9±2.0×10^4^	0.4	0.8	0.58
Urine Albumin Creatinine Ratio (mg/mmol)	3.4±0.4	13.2±1.5^##^	4.8±1.1^#^	0.0002	0.2	0.0006
Kidney/Body Weight Ratio (g/g)	6.9±0.2×10^−3^	9.5±0.4×10^−3ψ^	8.1±0.1×10−3*	<0.0001	0.01	0.009
24 hr Urine Volume (ml)	0.7±0.15	6.4±2.4^#^	3.9±1.6	0.005	0.06	0.21
Weight Gain (Fold change over original weight)	1.3±0.27	1.0±0.03^ψ^	1.2±0.05^#^	<0.0001	0.03	0.004
Blood Glucose level mmol/L	11.1±0.6	23.0±2.4^#^	21.1±3.2	0.0017	0.0001	0.33

### 9. Nox4 inhibition improves renal structure

In order to determine the effect of Nox4 inhibition on renal structure, kidneys from control and STZ-induced mice without and with plumbagin administration were immunostained by Periodic acid Schiff (PAS). Diabetic kidneys had increased mesangial matrix, mild glomerulosclerosis and increased tubular injury, characterised by separation of the tubules and tubular dilatation (Fig 9B) vs control (Fig 9A). In addition, STZ-induced mice have increased levels of proliferating cell nuclear antigen (PCNA) suggesting increased tubular cell proliferation (Fig 9E) vs control (Fig 9D). PAS and PCNA staining were reduced in diabetic mice administered with plumbagin (Fig 9 G and 9 H respectively).

**Figure 9:** Renal structure in diabetic mice in the presence and absence of Nox-4 inhibition. PAS staining (A, B,C) and immunohistochemistry for PCNA (D,E,F) showing that STZ-induced C57BL/6J mice have increased mesangial matrix, mild glomerulosclerosis and separation of tubules with tubular dilatation (B) in addition to increased proliferation (E) compared to control (A and D). Plumbagin (2 mg/kg/day) administration blocked diabetic induced effects (C and F). Proportion of area immunostained for PAS and PCNA is shown in (G and H) respectively. STZ and plumbagin were administered as described in the Material and Methods. Negative IgG was performed to confirm staining specificity (not shown). Magnification x 400.

### 10. Nox4 inhibition reduces TGF-β1, Fibronectin and CIV RNA expression in diabetic mice

In order to confirm the role of Nox4 inhibition *in vivo*, RNA was extracted from the three animal groups and real time PCR for fibronectin, collagen IV and TGF-β1 were determined. These results clearly demonstrate that diabetic mice express increased fibronectin, collagen IV and TGF-β1 mRNA to 1.5±0.1; 1.46±0.3 and 1.7±0.1 fold vs control respectively (all P<0.005) (Fig 10). Hence, not only were fibronectin and collagen IV significantly reduced in diabetic mice administered plumbagin, but interestingly, plumbagin inhibited the increased TGF-β1 expression in diabetic mice.

**Figure 10:** Expression of fibrotic markers in diabetic mice in the presence and absence of plumbagin. A) Fibronectin mRNA expression normalised to Actin. B) Normalized collagen IV mRNA expression, C) Normalized TGF-β1 mRNA expression. Results are expressed as mean ± SEM; n = 5–7. *#P*<0.005 and *P<0.05 vs. control or indicated experimental conditions.

### 11. Nox4 inhibition reduces extracellular matrix deposition induced by diabetes

The effect of Nox4 inhibition on renal fibrosis in the diabetic mouse model was determined by examining extracellular matrix deposition. Fibronectin immunohistochemistry and Masson Trichrome staining were used to determine extracellular matric expression. These results confirm that STZ-induced diabetic mice exhibit increased renal fibronectin and collagen IV deposition at 24 weeks post STZ induction (Fig 11B and 11E) vs control (11A and 11D), which was reduced with plumbagin administration (Fig 11C and 11F respectively).

**Figure 11:** Matrix deposition in diabetic mice in the presence and absence of Nox-4 inhibitor. Immunohistochemistry for fibronectin (A, B, C) and Masson Trichrome Staining (D,E,F) showing that STZ-induced diabetic C57BL/6J mice have increased fibronectin and collagen expression (B and E) respectively compared to control (A and D). Plumbagin (2 mg/kg/day) administration blocked diabetic induced effects (C and F). Proportion of area immunostained for fibronectin and collagen is shown in (G and H) respectively. STZ and plumbagin were administered as described in the Material and Methods. Negative IgG was performed to confirm staining specificity (not shown). Magnification x 400.

## Discussion

Diabetic nephropathy is the major cause of end-stage kidney failure throughout the world in both developed and emerging nations [21], [22]. It is functionally characterized by hyperfiltration and microalbuminuria, followed by a reduction in glomerular filtration rate and macroproteinuria [23], [24]. Pathologically there is excessive accumulation of extracellular matrix, thickening of glomerular and tubular basement membranes, increased mesangial matrix, loss of peritubular capillaries and vascular hypertrophy with a reduction in vessel luminal diameter. Early tubular injury has been reported in patients with diabetes mellitus whose glomerular function is intact [25] and tubulointerstitial injury has been recognized to correlate more closely than glomerular pathology with functional abnormalities [26], [27]. The epithelial cells of the proximal tubule are hence considered as major players in orchestrating renal interstitial fibrosis in diabetic nephropathy, with both hyperglycaemia [19], [20], [28], [29], [30], [31], [32], [33] and hypoxia [25], [34], [35], [36] considered to be the major initiators of cellular pathology.

It is widely accepted that although many factors are implicated in the cellular dysfunction observed in diabetes mellitus, high glucose-induced TGFβ1 [37], [38], [39], [40], [41], [42], [43] and its downstream signalling play an essential role in the development of renal fibrosis, indeed in all forms of nephropathy. Chronic hypoxia induces sequential abnormalities in oxygen metabolism including oxidative stress, nitrosative stress, advanced glycation, carbonyl and endoplasmic reticulum stress [44] in the kidneys of individuals with diabetes. Diabetic nephropathy is associated with a decrease of peritubular capillary number and hence reduced oxygen diffusion into the tubulointerstitial cells, leading to cellular hypoxia which ultimately contributes to renal fibrosis [25], [35], [45].

Nox4 is an NADP(H) oxidase that constitutively generates intracellular superoxide in the distal renal tubules [46], [47]. The exact physiological function of Nox4 has not yet been elucidated, but it may be an oxygen sensor that regulates erythropoietin production in the kidney. However, it has been implicated as a major source of renal ROS [48], [46]. Changes in cellular oxygen supply resulting in oxidative stress play an important role in the development and progression of diabetic nephropathy. Accumulating evidence also indicates that oxidative stress resulting in generation of ROS has a significant role in the initiation and progression of the ‘cardiorenal’ syndrome [49], [50]. Using rat kidney fibroblasts, Bondi et al. have demonstrated that TGF-β induces ROS production as part of its signal-transduction pathway [5]. The superoxide dismutase (SOD1) is the main isoform expressed in the kidney. It constitutes the first line of defence against ROS [51]. Since Nox4 is the major source of ROS in the kidneys during the early stages of diabetes, interventions to reduce ROS production by targeting Nox4 or increasing SOD1 may be an attractive therapeutic strategy.

Our study clearly demonstrates that high glucose and TGF-β1 increases Nox4 expression and TGF-β1 reduces SOD1 expression in human proximal tubule cells. In order to determine the role of Nox4 in TGF-β1 mediated renal fibrosis, two strategies to inhibit Nox4 were used, namely the administration of a Nox4 inhibitor in *in vitro* and *in vivo* studies and Nox4 specific siRNA in *in vitro* studies. Both approaches consistently and significantly reduce TGF-β1 induced fibronectin and collagen mRNA and protein expression, major extracellular matrix proteins that are upregulated in tubulointerstitial fibrosis. In keeping with our studies, Nox4 has been shown to play a role in liver and pulmonary fibrosis [52], [53]. Nox4 siRNA similarly reversed TGF-β1 effect on Nox4 and SOD1 expression suggesting a protective role against oxydative stress.

Using an STZ diabetes mouse model, we have demonstrated that Nox4 protein and ROS production are increased in the diabetic kidneys and their expression is largely localized to the tubules. Others have similarly demonstrated using *in situ* hybridization that Nox4 mRNA localizes in the renal cortex, specifically epithelial cells of proximal tubules, with lower expression in the medulla [48], [47].

Recent studies demonstrated that Nox4 may have protective effects [54], [55]. Using a Nox4 Knockdown mice model, Babelova et al. did not find evidence for a disease-promoting role of Nox4 but rather observed a small, yet significant protective effect against inflammation, fibrosis, and albuminuria [56] although characterizations of Nox4 knockout mice so far yielded no evidence for gross renal abnormalities [57], [58]. Zhang et al. found that Nox4 activity is regulated mainly by its expression level and Nox4-null animals developed exaggerated contractile dysfunction, hypertrophy, and cardiac dilatation during exposure to chronic overload whereas Nox4-transgenic mice were protected [57].

Nox4 was recently shown to be crucial for the survival of kidney tubular cells under injurious conditions. A protective role for Nox4 against kidney fibrosis during chronic renal injury was reported. The absence of Nox4 promoted kidney fibrosis with Nox4-deficient kidneys exhibiting increased oxidative stress [59]. On the other hand, Kleinschnitz et al. demonstrated that mice deficient in Nox4 (Nox4(–/–)) of either sex, but not those deficient for Nox1 or Nox2, were largely protected from oxidative stress, blood-brain-barrier leakage, and neuronal apoptosis, after both transient and permanent cerebral ischemia [58]. Interestingly, Schroder et al. has recently reported that endogenous Nox4 protects the vasculature during ischemic or inflammatory stress and hence low levels of Nox4 may have a protective vascular function [60]. Hence, it is biologically plausible that Nox4 plays a protective role under conditions where physiological levels of oxidative stress exist.

We have clearly demonstrated that Nox4 expression is upregulated in the diabetic kidney predominantly in areas of tubular pathology and that SOD1 expression is reduced. Administration of plumbagin preserved tubular architecture and this was associated with reduced expression of Nox4, increased expression of SOD1, increased activity of SOD and reduced expression of nitrotyrosine and 8-OHdG. It is recognised that no current pharmacological inhibitor, including plumbagin, is selective for Nox4 inhibition. However, our in vitro results, coupled with our in vitro data, suggest that elevated levels of TGFβ, as observed in diabetes, increases Nox4 expression that drives the development of tubulointerstitial pathology. The mechanism whereby Nox4 expression occurs with plumbagin administration is not clear. It is possible that diabetes induced ROS production is reduced by plumbagin and the downstream limitation in tubulointerstitial damage reduces Nox4 tissue expression. We have also demonstrated that administration of plumbagin significantly reverses diabetes induced upregulation of renal fibronectin and collagen IV mRNA and protein expression in the kidney. Furthermore increased mesangial expansion and tubular cell proliferation observed in the diabetic mice were reversed by treatment with plumbagin. It has been previously reported that cell proliferation increases in the tubulointerstitium, in contrast to glomerular cells in diabetic nephropathy [61].

Increased doses of plumbagin have been shown to induce toxicty [62], [63]. However, in the doses used in these studies, we have shown that 1μM of plumbagin has no toxic effect but is beneficial in reducing cell proliferation and cell damage induced with diabetes. A possible limitation of the present study is that a “plumbagin only” control group was not studied. However, the beneficial effect of plumbagin on PCNA expression, ROS markers and SOD expression and activity, suggest that a cytotoxic effect of plumbagin is very unlikely. In keeping with the diabetic phenotype, the diabetic C57BL/6J mice showed marked albuminuria elevated serum creatinine, and increased kidney/body weight. Importantly, plumbagin administration improved both physiological, and renal structural makers.

Our data collectively demonstrate a key role for plumbagin in diabetic induced fibrogenic responses in the kidney, with inhibition of TGFB induced Nox 4 activation being a target pathway.
